# Mammalian STE20-Like Kinase 2 Promotes Lipopolysaccharides-Mediated Cardiomyocyte Inflammation and Apoptosis by Enhancing Mitochondrial Fission

**DOI:** 10.3389/fphys.2020.00897

**Published:** 2020-08-06

**Authors:** Yanan Tian, Haijiu Song, Wei Qin, Zhenjiang Ding, Ying Zhang, Weichao Shan, Dapeng Jin

**Affiliations:** ^1^ Department of Cardiology, The Affiliated Hospital of Chengde Medical College, Chengde, China; ^2^ The First Department of Medicine, Chengde City Hospital of traditional Chinese Medicine, Chengde, China

**Keywords:** Mst2, inflammation, mitochondrial fission, cardiomyocyte, FCCP

## Abstract

In this study, we analyzed the role of mammalian STE20-like protein kinase 2 (Mst2), a serine-threonine protein kinase, in Lipopolysaccharides (LPS)-mediated inflammation and apoptosis in the H9C2 cardiomyocytes. Mst2 mRNA and protein levels were significantly upregulated in the LPS-treated H9C2 cardiomyocytes. LPS treatment induced expression of IL-2, IL-8, and MMP9 mRNA and proteins in the H9C2 cardiomyocytes, and this was accompanied by increased caspase-3/9 mediating H9C2 cardiomyocyte apoptosis. LPS treatment also increased mitochondrial reactive oxygen species (ROS) and the levels of antioxidant enzymes, such as GSH, SOD, and GPX, in the H9C2 cardiomyocytes. The LPS-treated H9C2 cardiomyocytes showed lower cellular ATP levels and mitochondrial state-3/4 respiration but increased mitochondrial fragmentation, including upregulation of the mitochondrial fission genes Drp1, Mff, and Fis1. LPS-induced inflammation, mitochondrial ROS, mitochondrial fission, and apoptosis were all significantly suppressed by pre-treating the H9C2 cardiomyocytes with the Mst2 inhibitor, XMU-MP1. However, the beneficial effects of Mst2 inhibition by XMU-MP1 were abolished by carbonyl cyanide-4-(trifluoromethoxy) phenylhydrazone (FCCP), a potent activator of mitochondrial fission. These findings demonstrate that Mst2 mediates LPS-induced cardiomyocyte inflammation and apoptosis by increasing mitochondrial fission.

## Introduction

Myocardial inflammation is the hallmark of several cardiovascular disorders, such as myocardial infarction, myocardial ischemia-reperfusion injury, diabetic cardiomyopathy, and sepsis-related myocardial damage (Gebhard et al., 2018; Zhong et al., 2019). The immune cells and pro-inflammatory cytokines involved in the inflammatory process promote cardiomyocyte dysfunction, which contributes to cardiovascular disease progression, severity, and outcomes (Ziegler, 2005). However, the molecular mechanisms underlying the inflammation-mediated cardiomyocyte dysfunction have not been fully understood.

Mitochondria play a central role in the regulation of cardiomyocyte viability and function (Wider et al., 2018). They are the main source of ATP production in the cardiomyocytes through oxidative phosphorylation and are essential for regulating cardiomyocyte contractility (Santin et al., 2019). Furthermore, damaged mitochondria induce cardiomyocyte death by triggering oxidative stress, ATP depletion, release of pro-apoptotic factors, and calcium overloading (Wang et al., 2019; Antonucci et al., 2020). Inflammation-related metabolic changes in the mitochondria have also been reported. Pirrozzi et al. (2020) reported that hepatic inflammation causes aberrant fatty acid metabolism in the mitochondria. The anti-inflammatory effects of omega-3 (DHA) in the neurodegenerative diseases are mediated by changes in mitochondrial functions (Braz-De-Melo et al., 2019). SIRT3 overexpression promotes mitochondrial function and attenuates vascular inflammation, endothelial dysfunction, vascular hypertrophy, and angiosteosis. Inflammation-related spinal cord injury (SCI) is caused by excessive production of mitochondrial reactive oxygen species (ROS). However, the relationship between mitochondrial dysfunction and inflammation-related cardiomyocyte damage has not been explored so far.

Mammalian STE20-like protein kinase 2 (Mst2) is a serine-threonine kinase that regulates tumor cell growth and survival. Mst2 regulates osteoblast differentiation by modulating Runx2 activity through phosphorylation (Won et al., 2019). Mst2 is essential for apoptosis of breast cancer cells and is associated with resistance against breast cancer therapy (Turunen et al., 2019). Several studies have also showed the association between Mst2 activation and mitochondrial dysfunction. Differential localization of A-Raf to the plasma membrane in epithelial cells releases Mst2, which then induces apoptosis by causing mitochondrial depolarization (Rauch et al., 2016). Mst2 also promotes mitochondrial ROS production in the phagocytes through the TLR-mediated assembly of the TRAF6-ECSIT complex in the mitochondria, which is essential for bactericidal activity (Geng et al., 2015). Mst2 activation is also involved in the adaptive response to inflammation. In vascular smooth muscle cells, Mst2 mediates miR-155-dependent inflammation and oxidative stress by altering the interaction between MEK and Raf-1(Yang et al., 2015). Genetic ablation of Mst2 attenuates inflammation-related hepatic injury (Kim et al., 2018). In cardiac diseases, cardiomyocyte dysfunction is related to inflammation that affects mitochondrial homeostasis (Silverblatt et al., 2019; Su et al., 2019). In this study, we aimed to understand the mechanistic role of Mst2 in inflammation-induced cardiomyocyte dysfunction using H9C2 cardiomyocytes as a model.

## Materials and Methods

### Cell Culture and Treatment

The H9C2 cardiomyocyte cell line was cultured in Dulbecco’s Modified Eagle’s medium (DMEM) (Nacalai Tesque Inc., Kyoto, Japan) containing 10% FBS, 100 μg/ml streptomycin, and 100 U/ml penicillin in a humidified chamber at 37°C in 5% CO_2_ as previously reported (Kim et al., 2019). The H9C2 cells were activated using 10 μg/ml Lipopolysaccharides (LPS) for 24 h. Mst2 activity was inhibited by incubating H9C2 cells with the Mst2 inhibitor XMU-MP1 (Cat. No. 6482, Bio-Techne China Co. Ltd.) for 6 h.

### Immunofluorescence Staining

LPS‐ or XMU-MP1-treated H9C2 cells were fixed with 4% paraformaldehyde for 10 min, washed with cold PBS three times, and blocked with 5% BSA in PBS on ice for 30 min. Then, the H9C2 cells were incubated overnight at 4°C with the primary antibody against TOM20 (1:1,000, Abcam, #ab186735). Then, after washing with cold PBS thrice, the cells were stained with Alexa Fluor-594 goat anti-mouse secondary antibody in 1% BSA/PBS for 1 h at 4°C. The cells were then permeabilized with 0.5% saponin for 15 min at room temperature, counterstained with DAPI, and the images were captured using a Nikon A1 confocal microscope (Wolint et al., 2019).

### Mitochondrial Membrane Potential

Mitochondrial membrane potential in H9C2 cells was determined using the JC-1 dye (Cat. No: C2006; Beyotime, China). In brief, the H9C2 cells were washed with PBS thrice, and then stained with JC-1 for 30 min in the dark. Then, the cells were washed thrice with PBS and images were captured using a Nikon A1 confocal microscope (van Duinen et al., 2019).

### Mitochondrial ROS Staining

We stained the H9C2 cells with Mitosox red, a mitochondrial superoxide-sensitive dye, as previously described (Aluja et al., 2019). In brief, H9C2 cells were washed thrice with PBS, and then stained with Mitosox red for 30 min in the dark. Then, after washing the cells with PBS, images were captured with the Nikon A1 confocal microscope.

### TUNEL Staining

H9C2 cells were incubated with the terminal deoxynucleotidyl transferase (TdT) enzyme and 2'-deoxyuridine 5'-triphosphate (dUTP) at 37°C for 1 h (Coverstone et al., 2018). Then, the nuclei was stained with 4',6-diamino-2-phenylindole (DAPI; Beyotime, C1006) for 5 min. The stained cells were photographed using a fluorescence microscope (Olympus FV3000RS) and the percentages of apoptotic cells were analyzed for each sample.

### MTT Assay

The MTT assay was performed as described previously. Briefly, we seeded 1 × 10^4^ H9C2 cells per well in 96-well plates overnight followed by incubation with LPS for 24 h. Then, after removing the medium, fresh medium supplemented with 0.5 mg/ml MTT (Solarbio) was added and the cells were cultured for another 4 h. The medium was then removed and the formazan product formed in the cells was extracted with 100 μl dimethyl sulfoxide (DMSO; Beyotime; Farber et al., 2018). The absorbance was read at 570 nm using a microplate reader (Enzyme-linked Biotechnology, Shanghai, China) and cell viability in the experimental group was normalized to the control (Rusnati et al., 2019).

### Quantitative Real Time PCR

Total RNA from H9C2 cells was isolated as previously described (Wolint et al., 2019) using the Quick-RNA MicroPrep kit (Zymo research). Then, 150–250 ng total RNA was reverse transcribed using the iScript cDNA synthesis kit (Bio-Rad). The cDNA samples were diluted 10-fold with ddH_2_O. Real-time quantitative PCR was performed using 2 μl cDNA from each sample in a LightCycler 480 (Roche). The relative mRNA expression was calculated using the 2^−ΔΔCt^ method with 18S RNA as an internal control (Dassanayaka et al., 2019).

### Statistics

The data are expressed as means ± SEM. Two-tailed student’s *t*-test was used to compare two groups and one-way or two-way ANOVA with Tukey’s test was used to compare multiple groups. *p* < 0.05 was considered statistically significant.

## Results

### Mst2 Promotes Inflammation in LPS-Treated H9C2 Cardiomyocytes

Mst2 gene expression was significantly higher in the LPS-treated H9C2 cells compared to the controls (Figure 1A). Immunofluorescence assays confirmed that Mst2 protein expression was significantly higher in the LPS-treated H9C2 cells compared to the controls (Figures 1B,C). These results demonstrate that LPS-mediated inflammation induces Mst2 mRNA and protein expression in H9C2 cardiomyocytes. Next, we tested if Mst2 is required for LPS-mediated inflammation in H9C2 cardiomyocytes by using the Mst2 inhibitor, XMU-MP1. Quantitative Real Time PCR (QRT-PCR) analysis showed that LPS-induced upregulation of IL-2, IL-8, and MMP9 mRNA levels in the H9C2 cardiomyocytes was blocked by pre-treatment with XMU-MP1 (Figures 1D–F). ELISA assay results confirmed that pre-treatment of H9C2 cardiomyocytes with XMU-MP1 blocked LPS-induced upregulation of IL-2, IL-8, and MMP9 protein levels (Figures 1G–I). These data demonstrate that Mst2 promotes LPS-mediated inflammation in H9C2 cardiomyocytes.

**Figure 1:** Mammalian STE20-like protein kinase 2 (Mst2) regulates inflammation in Lipopolysaccharides (LPS)-treated H9C2 cardiomyocytes. **(A)** Quantitative Real Time PCR (QRT-PCR) analysis shows Mst2 mRNA levels in the control and LPS-treated H9C2 cells. H9C2 cardiomyocytes were treated with LPS for 24 h. **(B,C)** Representative immunofluorescence images and quantitative analysis of Mst2 protein levels in the control and LPS-treated H9C2 cells. **(D–F)** QRT-PCR analysis shows IL-2, IL-8, and MMP9 mRNA levels in control, LPS-treated, and XMU-MP1 plus LPS-treated H9C2 cardiomyoctes. **(G–I)** ELISA assay results show IL-2, IL-8, and MMP9 levels in control, LPS-treated, and XMU-MP1 plus LPS-treated H9C2 cardiomyoctes. LPS treatment was performed for 24 h. H9C2 cells were pre-treated with the Mst2 blocker, XMU-MP1 for 6 h before treatment with LPS treatment. ^*^ *p* < 0.05.

### Mst2 Promotes Caspase-3/9-Mediated Apoptosis of LPS-Treated H9C2 Cardiomyocytes

Next, we analyzed the role of Mst2 in the apoptosis of LPS-treated H9C2 cardiomyocytes. MTT assay results show that LPS treatment significantly reduced the viability of H9C2 cells compared to the controls but pretreatment with XMU-MP1 attenuated apoptosis of LPS-treated H9C2 cells (Figure 2A). Moreover, the levels of LDH in the medium were significantly higher in LPS-treated H9C2 cells compared to controls but were reduced by pre-treatment with XMU-MP1 (Figure 2B). TUNEL staining assay showed that apoptotic rate was significantly higher in the LPS-treated H9C2 cells compared to the controls but was significantly reduced by XMU-MP1 pre-treatment (Figures 2C,D). These data suggest that Mst2 inhibition blocks LPS-mediated H9C2 cardiomyocyte apoptosis. We analyzed the levels of activated caspases-3 and caspases-9 to further understand the mechanism through which Mst2 mediates H9C2 cell death. The levels of activated caspase-3 and caspase-9 were significantly increased in LPS-treated H9C2 cells compared to the controls but were reduced by XMU-MP1 pre-treatment (Figures 2E,F). These results demonstrate that Mst2 promotes caspase-3/9-mediated apoptosis of LPS-treated H9C2 cardiomyocytes.

**Figure 2:** Mst2 promotes apoptosis of LPS-treated cardiomyocytes. **(A)** MTT assay results show the cell viability in the control, LPS-treated, and XMU-MP1 plus LPS-treated H9C2 cardiomyocytes. **(B)** LDH assay results show the levels of LDH in the growth medium of the control, LPS-treated, and XMU-MP1 plus LPS-treated H9C2 cardiomyocytes. **(C,D)** Representative TUNEL staining images and quantitative analysis of TUNEL-positive (apoptotic) cells in the control, LPS-treated, and XMU-MP1 plus LPS-treated H9C2 cardiomyocyte groups. **(E,F)** ELISA assay results show activated caspase-3 and caspase-9 levels in the control, LPS-treated, and XMU-MP1 plus LPS-treated H9C2 cardiomyocytes. LPS treatment was performed for 24 h. H9C2 cells were pre-treated with the Mst2 blocker, XMU-MP1 for 6 h before treatment with LPS treatment. ^*^ *p* < 0.05.

### Mst2 Regulates ATP Levels and Mitochondrial OXPHOS in LPS-Treated H9C2 Cardiomyocytes

Previous studies show that cardiac injury-related inflammation significantly alters mitochondrial structure and function (Kalyanaraman et al., 2018; Zhou et al., 2018a; Kowaltowski, 2019). Therefore, we analyzed if Mst2 alters mitochondrial structure and function in LPS-treated H9C2 cardiomyocytes. Mitochondrial membrane potential was significantly reduced in LPS-treated H9C2 cells compared to the controls but was higher in XMU-MP1 plus LPS-treated H9C2 cells (Figures 3A,B). Furthermore, mitochondrial ROS levels were higher in LPS-treated H9C2 cells compared to the controls but were lower in XMU-MP1 plus LPS-treated H9C2 cells (Figures 3C,D). The levels of antioxidant enzymes, such as GSH, SOD, and GPX, were also higher in LPS-treated H9C2 cells compared to the controls but were lower in the XMU-MP1 plus LPS-treated H9C2 cells (Figures 3E–G).

**Figure 3:** Mst2 mediates mitochondrial dysfunction in LPS-treated H9C2 cardiomyocytes. **(A,B)** FACS plots and quantitative analysis of JC-1 stained control, LPS-treated, and XMU-MP1 plus LPS-treated H9C2 cells are shown. Mitochondrial membrane potential was determined by evaluating the ratio of red-to-green JC-1 fluorescence intensity **(C,D)** Immunofluorescence analysis shows Mitosox red [mitochondrial reactive oxygen species (ROS)-sensitive dye] stained control, LPS-treated, and XMU-MP1 plus LPS-treated H9C2 cells. **(E–G)** ELISA analysis shows the levels of anti-oxidative proteins, namely, GSH, SOD, and GPX in the control, LPS-treated, and XMU-MP1 plus LPS-treated H9C2 cells. **(H)** The histogram shows ATP levels in the control, LPS-treated, and XMU-MP1 plus LPS-treated H9C2 cells. **(I,J)** Mitochondrial respiration assay results show the rate of state-3 and state-4 mitochondrial respiration in control, LPS-treated, and XMU-MP1 plus LPS-treated H9C2 cells. LPS treatment was performed for 24 h. H9C2 cells were pre-treated with the Mst2 blocker, XMU-MP1 for 6 h before treatment with LPS treatment. ^*^ *p* < 0.05.

Mitochondria are the major sites of ATP generation that is required for cardiomyocyte contractility (Liu et al., 2018a; Zhou et al., 2018b). Therefore, we analyzed if Mst2 regulates ATP levels and mitochondrial oxidative phosphorylation (OXPHOS) activities during LPS treatment of H9C2 cardiomyocytes. The ATP levels were significantly lower in the LPS-treated H9C2 cardiomyocytes compared to the controls but were higher in the XMU-MP1 plus LPS-treated H9C2 cells (Figure 3H). Moreover, mitochondrial state-3 and state-4 respiration rates were reduced in LPS-treated H9C2 cells but were higher in XMU-MP1 plus LPS-treated H9C2 cells (Figures 3I,J). These data demonstrate Mst2 regulates ATP levels and mitochondrial OXPHOS in LPS-treated H9C2 cardiomyocytes.

### Mst2 Promotes Mitochondrial Fission in LPS-Treated H9C2 Cardiomyocytes

Since excessive mitochondrial fission is linked to mitochondrial dysfunction (Fuhrmann et al., 2019; Wang et al., 2020b), we tested if Mst2 promotes mitochondrial fission in LPS-treated H9C2 cardiomyocytes. QRT-PCR analysis showed that the mRNA levels of Drp1, Mff, and Fis1 (mitochondrial fission-related proteins) were significantly higher in LPS-treated H9C2 cells compared to the controls but were significantly lower in the XMU-MP1 plus LPS-treated H9C2 cells (Figures 4A–C). Immunofluorescence analysis showed that the number of fragmented mitochondria were significantly higher in LPS-treated H9C2 cells compared to the controls but were significantly lower in the XMU-MP1 plus LPS-treated H9C2 cells (Figures 4D,E). These data demonstrate that Mst2 promotes mitochondrial fission in LPS-treated H9C2 cardiomyocytes.

**Figure 4:** Mst2 induces excessive mitochondrial fission in LPS-treated H9C2 cardiomyocytes. **(A–C)** QRT-PCR analysis shows Drp1, Mff, and Fis1 levels in the control, LPS-treated, and XMU-MP1 plus LPS-treated H9C2 cells. **(D,E)** Representative immunofluorescence images show Alexafluor-594-tagged-anti-TOM20 antibody-stained control, LPS-treated, and XMU-MP1 plus LPS-treated H9C2 cells. Also shown is the quantification of the ratio of fragmented mitochondria in control, LPS-treated, and XMU-MP1 plus LPS-treated H9C2 cell groups. LPS treatment was performed for 24 h. H9C2 cells were pre-treated with the Mst2 blocker, XMU-MP1 for 6 h before treatment with LPS treatment. ^*^ *p* < 0.05.

### Re-activation of Mitochondrial Fission Abolishes Mst2 Inhibition-Mediated Mitochondrial Protection and Cardiomyocyte Survival

Next, we analyzed if carbonyl cyanide-4-(trifluoromethoxy)phenylhydrazone (FCCP), an activator of mitochondrial fission, induces mitochondrial fragmentation, mitochondrial dysfunction, and apoptosis in the XMU-MP1 plus LPS-treated H9C2 cells. MTT assay results showed that FCCP treatment significantly reduced the viability of the XMU-MP1+LPS-treated H9C2 cardiomyocytes (Figure 5A). Furthermore, FCCP treatment significantly increased the percentage of TUNEL-positive cells in the XMU-MP1+LPS-treated H9C2 cardiomyocytes (Figures 5B,C). Furthermore, FCCP treatment significantly increased mitochondrial ROS in the XMU-MP1+LPS-treated H9C2 cardiomyocytes (Figures 5D,E). FCCP treatment also reduced the levels of antioxidant enzymes, GSH, SOD, and GPX in the XMU-MP1+LPS-treated H9C2 cardiomyocytes (Figures 5F–H). These results confirm that Mst2 promotes LPS-induced H9C2 cardiomyocyte apoptosis by increasing mitochondrial fission.

**Figure 5:** Carbonyl cyanide-4-(trifluoromethoxy) phenylhydrazone (FCCP) re-activates mitochondrial fission and abolishes the cardiomyocyte protective effects of the Mst2 inhibitor. **(A)** MTT assay results show the viability of control, LPS-treated, XMU-MP1 plus LPS-treated, and FCCP plus XMU-MP1 plus LPS-treated H9C2 cells. **(B,C)** TUNEL staining images and quantification of percent TUNEL+ (apoptotic) cells in the control, LPS-treated, XMU-MP1 plus LPS-treated, and FCCP plus XMU-MP1 plus LPS-treated H9C2 cardiomyocyte groups are shown. **(D,E)** Immunofluorescence analysis shows the Mitosox red (mitochondrial ROS-sensitive dye)-stained control, LPS-treated, XMU-MP1 plus LPS-treated, and FCCP plus XMU-MP1 plus LPS-treated H9C2 cardiomyocyte groups. **(F–H)** ELISA assay results show the levels of antioxidant enzymes, namely, GSH, SOD, and GPX in the control, LPS-treated, XMU-MP1 plus LPS-treated, and FCCP plus XMU-MP1 plus LPS-treated H9C2 cardiomyocyte groups. Cardiomyocytes were treated with LPS for 24 h. Mst2 blocker (XMU-MP1) was used to incubate with cardiomyocyte before LPS treatment. FCCP was used to increase mitochondrial fission. ^*^ *p* < 0.05.

## Discussion

In this study, we explored the role of Mst2 in LPS-induced cardiomyocyte inflammation and apoptosis. Our data demonstrates that Mst2 mRNA and protein expression is significantly upregulated in LPS-treated cardiomyocytes. Moreover, Mst2 promotes cardiomyocyte inflammation and triggers apoptosis. Mst2 activation increases mitochondrial fission, mitochondrial ROS, mitochondrial OXPHOS dysfunction, and oxidative stress. Mst2 inhibition by XMU-MP1 attenuates LPS-mediated cardiomyocyte apoptosis and mitochondrial dysfunction partly through the inhibition of mitochondrial fission. However, re-activation of mitochondrial fission through FCCP abolishes the beneficial effects of Mst2 inhibition. By our knowledge, this is the first study to describe the role of Mst2 in inflammation-related cardiomyocyte dysfunction and apoptosis.

Several studies show that inflammation plays a significant role in cardiovascular disorders, such as atherosclerosis, hypertension, post-infarction myocardial remodeling, acute ischemia-reperfusion injury, and atrial fibrillation (Cuadrado et al., 2018; Gaspar et al., 2018). Several molecular mechanisms have been proposed to explain the influence of inflammation on cardiovascular disorders (Battistelli et al., 2019; Song and Li, 2019), including the formation of the NLRP3 inflammasome, which induces endothelial cell dysfunction and accelerates the progression of diabetes-related atherosclerosis (Eid et al., 2018; Zheng et al., 2019). In mice with diet-induced obesity, endothelial anticoagulant mechanism is impaired by inflammation and is accompanied by the vascular calcification (Aguilar et al., 2019; Zhang et al., 2019b). Pulmonary arterial hypertension is associated with systemic inflammation (Ntiloudi et al., 2019; Zhang et al., 2019a). Several anti-inflammatory drugs have been developed to suppress inflammation in cardiovascular disorders. This includes a hydrogen sulfide donor, GYY4137, which suppresses inflammasome activation and protects against diabetes-induced atherosclerosis (Trindade et al., 2019; Zheng et al., 2019). Kuzewski et al. (2020) reported that fish oil and curcumin supplementation reduces the serum levels of pro-inflammatory biomarkers and improves cerebrovascular function in older adults. Melatonin, a hormone that regulates the sleep-wake cycle, suppresses post-infarction myocardial inflammation and attenuates cardiac remodeling (Liu et al., 2018b; Morell et al., 2018; Liang and Huang, 2019). Although our study demonstrates that Mst2 is a novel regulator of inflammation-related cardiomyocyte viability, further investigations are necessary to determine the therapeutic potential of targeting Mst2 in cardiovascular diseases.

Our data shows that Mst2 promotes LPS-mediated cardiomyocyte dysfunction by inducing mitochondrial fission. Under normal conditions, mitochondrial fission is required for mitochondrial proliferation, mitochondrial distribution during cell division, and segregating damaged mitochondria from functional mitochondria to maintain mitochondrial function and quality (Paul et al., 2018; Qaisar et al., 2019). In disease conditions, excessive mitochondrial fission decreases mitochondrial membrane potential and respiratory functions (Cabon et al., 2018; Walraven et al., 2018). Excessive mitochondrial fission is implicated in cardiomyocyte dysfunction and/or death (Wang et al., 2018; Kowaltowski, 2019). Abnormal mitochondrial fission is associated with opening of the mitochondrial permeability transition pore (mPTP), which results in reduction of the mitochondrial membrane potential and induction of caspase-9-related apoptotic pathway (Lim and Murthy, 2018; Linkermann, 2019). Besides, mitochondrial fission promotes the expression of pro-inflammatory factors, such as ICAM-1 or ET-1, thereby contributing to endothelial dysfunction and cardiovascular dysfunction (Zhou et al., 2018a). Zhou et al. (2019) firstly reported that mitochondrial fission plays a central role in the pathogenesis of inflammation-related hepatic disorders, such as alcoholic liver damage and fatty liver disease, by decreasing hepatocyte glucose metabolism and promoting fatty acid accumulation in the liver tissues. Mitochondrial quality control mechanisms including mitochondrial fission play a central role in acute cardiac injury (Wang et al., 2020a,b).

In conclusion, our study demonstrates that Mst2 is a novel regulator of mitochondrial fission and apoptosis in inflammation-related cardiomyocyte dysfunction.

## Data Availability Statement

All datasets presented in this study are included in the article/supplementary material.

## Author Contributions

YT contributed to the study concepts, study design, data acquisition, and manuscript preparation. HS and WQ contributed to study concepts, study design, literature research, data acquisition, manuscript preparation, and editing. YT and ZD were the guarantors of integrity of the entire study and contributed to statistical analysis and manuscript review. YZ, WS, and DJ contributed to experimental studies and data acquisition. All authors contributed to the article and approved the submitted version.

### Conflict of Interest

The authors declare that the research was conducted in the absence of any commercial or financial relationships that could be construed as a potential conflict of interest.
